The article "Aging-associated distinctive DNA methylation changes of LINE-1 retrotransposons in pure cell-free DNA from human blood" was retracted in 2022. Reasons: duplicated images; original data or images not available.

# Aging-associated distinctive DNA methylation changes of LINE-1 retrotransposons in pure cell-free DNA from human blood

**DOI:** 10.1038/s41598-020-79126-z

**Published:** 2020-12-17

**Authors:** Wardah Mahmood, Lars Erichsen, Pauline Ott, Wolfgang A. Schulz, Johannes C. Fischer, Marcos J. Arauzo-Bravo, Marcelo L. Bendhack, Mohamed Hassan, Simeon Santourlidis

**Affiliations:** 1 Epigenetics Core Laboratory, Institute of Transplantation Diagnostics and Cell Therapeutics, Medical Faculty, Heinrich-Heine University Duesseldorf, Moorenstr. 5, 40225 Duesseldorf, Germany; 2 Department of Urology, Medical Faculty, Heinrich-Heine University, Duesseldorf, Germany; 3 Institute of Transplantation Diagnostics and Cell Therapeutics, Medical Faculty, Heinrich-Heine University Duesseldorf, Moorenstr. 5, 40225 Duesseldorf, Germany; 4 Group of Computational Biology and Systems Biomedicine, Biodonostia Health Research Institute, 20014 San Sebastián, Spain; 5 IKERBASQUE, Basque Foundation for Science, 48009 Bilbao, Spain; 6 Department of Urology, University Hospital, Positivo University, Curitiba, Brazil; 7 Department of Surgery, Tulane University School of Medicine, New Orleans, LA 70112 USA; 8 Institut National de La Santé Et de La Recherche Médicale, University of Strasbourg, 67000 Strasbourg, France

**Keywords:** Cell biology, Molecular medicine

## Abstract

LINE-1 hypomethylation of cell-free DNA has been described as an epigenetic biomarker of human aging. However, in the past, insufficient differentiation between cellular and cell-free DNA may have confounded analyses of genome-wide methylation levels in aging cells. Here we present a new methodological strategy to properly and unambiguously extract DNA methylation patterns of repetitive, as well as single genetic loci from pure cell-free DNA from peripheral blood. Since this nucleic acid fraction originates mainly in apoptotic, senescent and cancerous cells, this approach allows efficient analysis of aged and cancerous cell-specific DNA methylation patterns for diagnostic and prognostic purposes. Using this methodology, we observe a significant age-associated erosion of LINE-1 methylation in cfDNA suggesting that the threshold of hypomethylation sufficient for relevant LINE-1 activation and consequential harmful retrotransposition might be reached at higher age. We speculate that this process might contribute to making aging the main risk factor for many cancers.

## Introduction

Each year, over 9 million people die from cancer worldwide^1^, despite continuous progress in treatment and therapy. This high mortality could be reduced by appropriate diagnostic procedures applied in the long periods during which cancers at treatable stages remain concealed. In various cancer types, e.g. ovarian, lung, pancreatic, colorectal, and breast carcinoma as well as melanoma, early diagnosis at a localized stage is associated with a significantly increased 5-years survival rate in comparison to metastatic disease, at which cancer is too often diagnosed^2^. Evidently, sensitive and specific biomarkers for early diagnosis, prognosis and monitoring could relieve this unfortunate state, saving lives and reducing morbidity. One new approach at providing such biomarkers combines epigenetics with liquid biopsies.

Liquid biopsies, i.e., the analysis of cell-free DNA (cfDNA) from a minimal-invasive routine blood draw or a urine sample, are convenient, cost-effective and patient-friendly. Normally, cfDNA of peripheral blood is a small, free-floating, strongly fragmented nucleic acid fraction with major average lengths of ~ 170 bp, ~ 340 and 510 bp. These sizes correspond to the length of DNA wrapped around one, two or three nucleosomes^3^. It is thought that this nucleosomal fragmentation profile is due to the preferential cleavage of internucleosomal linker DNA during apoptotis^4^. In healthy donors cfDNA is released by a combination of apoptosis, necrosis, and secretion to a concentration not exceeding 5–10 ng/ml^3^. It is derived from white blood cells (55%), erythrocyte progenitors (30%), vascular endothelial cells (10%) and hepatocytes (1%), with plasma of older people showing significantly higher levels of total cfDNA^5^. CfDNA has a half-life of less than 2 h^6,7^. In cancer, additional cfDNA is released by apoptosis or necrosis or is shed by viable tumor cells^8^ so that the total cfDNA concentration may increase by up to 50-fold compared to healthy persons, depending on the type of cancer and the burden of disease^3^. Noteworthy, total cfDNA levels were observed to decrease after therapy or surgery^8^.

The methylome consists of all methylated cytosine-guanosine (CpG) dinucleotides of the genome, forming an elaborate, plastic and cell-type specific molecular pattern that determines genome organization, gene regulation and thereby cellular phenotype and function. Furthermore, DNA methylation preserves genome integrity by repressing transposable genetic elements^9^. Stable cancer cell-specific DNA methylation alterations occur during early steps of the carcinogenesis process and are ideal for sensitive, rapid and cost-effective detection by techniques like methylation-specific PCR^8^. Methylation patterns can moreover predict prognosis and survival^10^. Importantly, certain aberrant DNA methylation patterns are found across different cancer types making them suitable for a “PANCancer” diagnosis, i.e., simultaneous screening for several cancer types in one approach^11^. Since tumors shed cfDNA^3^, cancer cell-specific DNA methylation signatures in cfDNA allow identification of breast, colon and lung cancer, e.g.^5^. A plethora of data indicate that even patient stratification by prognosis, recurrence risk and response to therapy can be achieved by analyzing gene methylation signatures on cfDNA extracted from plasma or serum^11^.

LINE-1 hypomethylation, a loss of DNA methylation in the CpG-rich promoter sequences of Long Interspersed Nuclear Elements retrotransposons, occurs as “genome-wide” or “global” DNA hypomethylation in many cancer types, including colon, lung, prostate and breast cancer, hepatocellular and gastric carcinoma, and chronic lymphocytic leukemia (CLL). LINE-1 hypomethylation is therefore one of the characteristic methylation profile changes common to many cancers^12–14^. LINE-1 hypomethylation often leads to LINE-1 activation^12^, i.e., expression of LINE-1 RNA and proteins, including its potent endonuclease. This activation may elicit DNA damage and repair, stress responses, tumor progression and apoptosis, especially if additional cellular retrotransposition control mechanisms have been overcome^13^.

For instance, we have recently shown that interference with methyl group availability by downregulation of ornithine decarboxylase, a key enzyme of polyamine biosynthesis, can induce LINE-1 hypomethylation in primary uroepithelial cells, leading to increased LINE-1 transcript levels, double-strand DNA breaks and decreased viability^15^.

Interestingly, a gradual loss of LINE-1 methylation has also been observed during aging that may likewise derepress silenced LINE-1 retroelements followed by increased genomic instability^16^. Aging is known as a main risk factor for cancer. In this regard, we had provided additional evidence that genome-wide hypomethylation of LINE-1 retroelements in cfDNA in blood is an epigenetic biomarker of human aging^17^. Recently, it has been shown that LINE-1 sequences are a major component of circulating cfDNA^18^. This finding suggests the idea that cfDNA may originate in aging or tumor cells afflicted by LINE-1 hypomethylation. Such cells would have a significantly elevated rate of LINE-1 activation and retrotransposition, affecting genomic integrity. Ultimately, this could result in apoptosis and release of their LINE-1-enriched cfDNA. In support of this inference, genomic instability has been implicated as a cause of aging since the late 1940s^19^ and is recognized as a hallmark of cancer^20^.

DNA methylation patterns of cfDNA in peripheral blood are thus of central importance for aging research and cancer diagnosis, prognosis and monitoring, but also for elucidating the epigenetic component making aging a main risk factor for cancer.

Here, we first present a simple but effective methodological approach to unambiguously uncover detailed DNA methylation patterns from cfDNA, i.e., for every single CpG dinucleotide position, either from repetitive or any single genomic segment of interest. We have previously demonstrated that the knowledge on detailed cancer type-specific DNA methylation patterns for every relevant CpG dinucleotide position is essential for the design of MS-PCR primers to identify cancers and maximize diagnostic efficiency^21^. In addition, to accurately measure DNA methylation differences in samples with varying numbers of target loci due to genome instability, we have developed the technique of idiolocal normalized real-time methylation-specific PCR (IDLN-MSP)^22^. Noteworthy, it has been shown that the frequency of genome rearrangements increases with age^23^. Especially age-dependent aneuploidy, i.e. the loss or gain of whole chromosomes, was first described for human lymphocytes^24^.

Our approach presented here provides cfDNA completely free of DNA contamination from blood cells, which have their own specific methylation pattern and might therefore mask the pattern from cfDNA. We then exemplarily compare the detailed cfDNA LINE-1 methylation pattern from peripheral blood of young and aged individuals revealing a significant difference.

## Results

### Age correlated decrease of LINE-1 retrotransposon promoter methylation in cell-free DNA of peripheral blood

To extend our previous evidence on LINE-1 retrotransposon hypomethylation as a biomarker for human aging^17^, we optimized the isolation procedure of cfDNA as described in detail in the Materials & Methods section. In brief, we comparatively tested four different commercial kits for isolation of cfDNA. In our hands only one product reproducibly delivered cfDNA without visible cellular DNA contamination (Fig. 5). Nevertheless, after intensively interrogating the product representatives in no case they weren’t able to definitely assure that co-isolation of residual cellular DNA can be excluded. In contrast one of them showed us own comparative inter-company analyses documenting residual signals of cellular DNA contaminations.

Using this established, cleaner separation of circulating cfDNA from the DNA of blood cells, we quantified LINE-1 retrotransposon promoter methylation in both DNA fractions. Healthy donors from the German general population without pre-existing conditions, aged between 19 and 73, provided blood samples. LINE-1 methylation was measured by Idiolocal Normalized real-time Methylation-Specific PCR (IDLN-MSP), which improves the accuracy of relative quantification by intercalating dye real-time MSP in DNA samples that may harbor genetic imbalances^22^. Notably, the frequency of genome rearrangements increases with age^19^. Primers for MSP were optimized based on bisulfite sequencing as described below in “Age-dependent distinct erosion of LINE-1 promoter methylation in cell-free DNA of peripheral blood” section.

Relative to the mean value of samples from two individuals aged 19 and 22 years set as 1, relative DNA methylation levels in the other samples ranged from 0.81 to 1.97 in cellular DNA and from 0.16 to 2.88 in cfDNA (Fig. 1A/C). LINE-1 DNA methylation in cellular DNA remained relatively stable with age, with no apparent increase or decrease (Pearson’s correlation coefficient R^2^ = 0.01). In contrast LINE-1 DNA methylation in cfDNA decreased with age (Pearson’s correlation coefficient R^2^ = 0.31). The decline in cfDNA methylation was accentuated if sample cohorts were stratified according to gender or quartiles by age (19–30, 31–40, 41–50 and 51–60 years; 19–30 to 31–40, p = 0.01, 19–30 to 41–50, p = 0.0000043026, 19–30 to 51–60, p = 0.0000000049, 31–40 to 41–50, p = 0.1897896039, 31–40 to 51–60, p = 0.0040846031) (Fig. 1D). In comparison, cellular DNA methylation tends to be higher in females than males in the age groups between 19 and 40 years; this tendency becomes reversed in the 41–50 years subgroup (Fig. 1B). In cfDNA methylation, no gender differences were observed. Thus, DNA methylation of the LINE-1 promoter region remains stable in both genders during aging in the DNA of peripheral blood cells but decreases with age in cfDNA from peripheral blood of both genders.

**Figure 1:** Relative quantification of age-dependent LINE-1 methylation by IDLN-MSP in cellular and cfDNA. Correlation between age and DNA methylation of LINE-1 promoter region in cellular DNA (**A**, **B**) and cell-free DNA (**C**, **D**) derived from blood plasma of the indicated numbers of donors (N). The regression lines are colored in red and represent Pearson’s correlation coefficients (R^2^). Mean values of global DNA methylation at LINE-1 retrotransposons in cellular DNA and cell-free DNA from blood plasma by age subgroups (**B**, **D**). Mean values were compared by two-sample Student’s t-test with a significance threshold p < 0.05. 19–30 to 31–40 years, p = 0.01, 19–30 to 41–50 years, p = 0.0000043026, 19–30 to 51–60 years, p = 0.0000000049, 31–40 to 41–50 years, p = 0.1897896039, 31–40 to 51–60 years, p = 0.0040846031, 1D).

### Age-dependent distinct erosion of LINE-1 promoter methylation in cell-free DNA of peripheral blood

To follow up on this finding we analyzed the DNA methylation patterns of the promoter region of LINE-1 retrotransposons in cfDNA in detail by bisulfite sequencing using a previously described procedure^21^. A prerequisite for this is the availability of pure cell-free DNA without residual contaminations by cellular DNA. Therefore, we did not rely on the commercial kit and followed a new strategy. This strategy relies on the fact that contaminating cellular DNA liberated during preparation from blood cells is larger in size, whereas cfDNA is known to consist of a major fraction with an average length of ~ 170 bp corresponding to the length of DNA wrapped around one nucleosome plus a linker sequence^7^ and further fractions of multiple length of ~ 340 bp, ~ 510 bp and ~ 680 bp in decreasing quantities^3^. These sizes are thought to be generated by the action of caspase-activated endonucleases that cleave DNA between nucleosomes during apoptosis, a major source of cfDNA release^26^. Therefore, excision of DNA of these sizes following agarose gel electrophoresis will strongly enrich for cfDNA. Since the total amount of cfDNA in circulating blood of healthy individuals is very low, typically around 5 to 10 ng/ml, it cannot be visualized by ethidium bromide staining. In addition, DNA is further degraded by bisulfite treatment. Therefore, it is widely assumed that this electrophoretically separated, invisible cfDNA fraction should defy further analytical epigenetic analyses, e.g. bisulfite sequencing.

Indeed, DNA from cfDNA preparations was not visible in gels (Fig. 2A/B), but we could obtain unambiguous LINE-1 promoter amplification products from the material blindly excised by size (Fig. 2C, suppl. Fig. 1). We assume that the natural fragmentation of cell-free DNA as for instance has been visualized by Jahr et al. with silver staining in polyacrylamide gels^27^ consists a further supportive parameter of template amenability for efficient MSPCR. Next, we performed MS-PCR on the extracted and bisulfite-treated cfDNA for the single diploid locus *OR52J3* and obtained amplification products (Fig. 2D, suppl. Fig. 1), although only after nested amplification. Hence, although fragmented cfDNA persists in low amounts in peripheral blood of healthy individuals, undetectable by conventional ethidium bromide staining, it can be isolated in a pure form from conventional agarose gels after separation and MS-PCR amplifications, the bottleneck of subsequent bisulfite sequencing, are unreservedly amenable from repetitive as well as single genetic spots.

**Figure 2:** Excision of invisible cfDNA and MSPCR amplification of repetitive and single genomic segments. CfDNA and cellular DNA (gDNA) isolated from young and older individuals were excised from agarose gels after electrophoretic separation (**A**/**B**), bisulfite treated, and LINE-1 and *OR52J3* promoter amplification products were generated (**C**/**D**).

Next, we applied bisulfite sequencing to cellular and cell-free DNA of 8 young (21–29 years) and 8 older (50–58 years) individuals, combining the each 8 samples for analysis. This method is technically independent of MS-PCR in so far as the primers do not cover and bind differentially methylated CpG positions to interrogate their methylation status but bind to CpG free sequences surrounding CpG-rich DNA sequences. Sequencing of the amplified fragments allows to uncover the methylation status of every enclosed CpG-position. Using this method, we found different DNA methylation levels in cellular DNA, with 62% and 50% methylation in young and old individuals, respectively (Fig. 3A), but these differences were much more pronounced in cfDNA from the same individuals, with 68% and 20% methylation in young and old individuals, respectively (Fig. 3B). Thus, cfDNA methylation of LINE-1 retrotransposon promoters in healthy elder individuals is eroded in comparison to their cellular DNA and to the cfDNA of young individuals. In particular, hypomethylation affects completely unmethylated sequences matching closely (97–98%) to known full-length LINE-1 sequences with intact open reading frames (sequences kindly provided by Dr. Goodier, Johns Hopkins University School of Medicine). It has been shown that at least 100 full-length LINE-1 elements of the human genome are capable of retrotransposition and their mobilization is associated with genomic instability^28^. The most strongly age-dependent methylation changes in cfDNA occur at CpG positions -29, -27, -23, -20, -17, -14, and -13 (Fig. 3C). Taking this information into account together with the required thermodynamic parameters we chose primers for MS-PCR to cover CpG -27 to -24 (upper primer) and -15 to -14 (lower primer) in order to achieve optimal discrimination and accuracy for subsequent IDLN-MSPCR to study age-dependency of methylation in cell-free DNA (Fig. 1).

**Figure 3:** Detailed analysis of LINE-1 promoter CpG-methylation derived from peripheral blood cellular DNA (**A**) and cell-free DNA (**B**) of 8 young individuals aged 21–29 years (left panels) and 8 elder individuals aged 50–58 years (right panels). On top, a schematic representation of a full-length LINE-1 retroelement is given showing the distribution of CpG dinucleotides (short vertical lines) and the open reading frames 1 and 2 (ORF1/2). The analyzed 436 bp region of interest is indicated by square brackets. Detailed CpG-methylation profiles of this region revealed by bisulfite genomic sequencing are shown in panels A and B. Filled circles stand for methylated CpG dinucleotides. White circles stand for unmethylated CpGs. Grey circles stand for an undefined CpG methylation status. In the panel C the result is illustrated in bar diagrams in order to visualize the most differentially methylated CpG positions. Each bar shows the frequency of methylated CpGs at the position indicated. Positions are relative to the ATG start codon of LINE-1 ORF1. An asterisk indicates the positions of the primers used for the MS-PCR shown in Fig. 1. The left diagram shows the analyses from peripheral blood cellular DNA of young (green) and elder (blue) individuals. The right diagram shows the analyses from peripheral blood cfDNA of young (green) and elder (blue) individuals.

### LINE-1 ORF1p is not detectable in peripheral blood of healthy individuals

It is widely accepted that DNA methylation represses repetitive DNA elements including LINE-1 retrotransposons to ensure genomic integrity, its stability and to prevent cancer. LINE-1 hypomethylation seems to be a sufficient criterion for LINE-1 transcription, as demonstrated by us and others^15^. However, additional potent mechanisms in healthy somatic cells inhibit LINE-1 protein expression. The LINE-1 ORF1p and ORF2p proteins are parts of an efficient endonuclease-driven retrotransposition machinery which is active in many cancers and correlates with LINE-1 insertion mutagenesis and genomic instability^29^. To determine whether the marked hypomethylation of the LINE-1 promoter in cfDNA leads to detectable protein expression in peripheral blood, we established a sensitive ELISA assay for LINE-1 ORF1p. ORF1p was chosen as a target, because it is expressed at much higher levels than ORF2p^30^. As a positive control, the expression of ORF1p was well detectable in HT-1376 urothelial cancer cells. However, despite repeated attempts we could neither detect a significant higher signal for LINE-1 ORF1p in peripheral blood plasma of individuals aged between 58–63 years nor individuals aged 19–23 years (Fig. 4).

**Figure 4:** ELISA analysis of LINE-1 ORF-1 product on peripheral blood of young and older individuals. Cell lysate from the urothelial bladder cancer cell line HT1376 and primary urothelium were used together with water and blood plasma from young and older individuals.

## Discussion

DNA methylation signatures from the cfDNA of body fluids are increasingly gaining interest for diagnosis, prognosis and monitoring of a broad spectrum of major diseases and to study epigenetic deterioration, caused, e.g., by aging or lifestyle. The exploitation of epigenetic features of cfDNA has the potential to contribute to significant reductions of mortality and morbidity and to the improvement of quality of life. However, before reliable routine applications on patients can come into practice, many details have still to be worked out.

For instance, in previous studies conflicting results have been obtained on the association of age with Alu and LINE-1 methylation^31^. On the one hand, a study that used blood samples from 718 elderly male subjects between 55 and 92 years reported that Alu methylation decreased during aging whereas LINE-1 methylation did not vary over time^31^. Similarly, Jintaridth et al. observed age-dependent hypomethylation of Alu and HERV-K, but not hypomethylation of LINE-1 in peripheral blood mononuclear cells^32^. On the other hand, it has been reported that LINE-1 sequences become demethylated with age in white blood cells, while smoking and drinking have no significant effect on LINE-1 hypomethylation^33^. In our own previous study, we found LINE-1 hypomethylation in cell-free DNA, but not in cellular DNA from peripheral blood to constitute an epigenetic biomarker for human aging and we described more extensive changes in smokers^17^. We suggest that these discrepancies might be due, at least partly, to the technical issue that it is difficult to obtain cfDNA completely free of cellular DNA contamination and therefore, contaminating cellular DNA with its own distinct DNA methylation pattern may confound the cfDNA patterns. Indeed, when testing a variety of commercial cfDNA isolation kits we found almost universally residual cellular DNA contamination. Ultimately, in our hands only one kit reproducibly yielded no visible cellular DNA contamination, at least at the sensitivity of ethidium bromide-stained agarose gels. Applying a new purification technique based on excision of cfDNA bands from agarose gels we demonstrate here a clear correlation between increasing LINE-1 hypomethylation in cfDNA and age for both genders, whereas methylation of cellular DNA was relative stable in individuals between 19 and 73 years. This observation appears in accordance with the notion that the cellular DNA belongs to highly differentiated and functionally specialized but relative short living leukocytes, i.e. neutrophils, lymphocytes, monocytes, eosinophils and basophils that have life spans from a few hours to weeks^34^. These cells are continuously replaced by new ones by the constitutively robust functioning hematopoietic system of people of young, middle and higher age. However, further studies should be made to clarify whether cellular DNA LINE-1 methylation declines at advanced age, i.e. beyond 70 years, where hematopoiesis often declines. Noteworthy, after splitting in several age subgroups we found a minor reduction of methylation in females aged 41–50 years, i.e. approaching menopause, in cellular DNA as was previously described by others^35^. Our finding therefore supports the conclusion of these authors that altered DNA methylation in leukocytes and serum cell-free DNA may represent a biomarker of approaching menopausal age.

As an alternative technique for specific enrichment of cfDNA, we applied agarose gel electrophoresis as an effective way of separating DNA fragments of varying sizes^36^. The oligo-nucleosomal pattern of cfDNA is well described and has especially been demonstrated by silver staining in polyacrylamide gels after electrophoretic separation^37^. Therefore, excising the appropriate part of the agarose gel yields predominantly cfDNA, even though it is not visible following ethidium bromide staining. We assumed that both the fragmentation pattern of cfDNA and the repetitive nature of LINE-1 elements favor the generation of amplicons from such very low amounts of cfDNA even after bisulfite treatment, which can lead to significant DNA degradation. However, we showed that even a diploid sequence in the genome like *OR52J3* can be amplified by nested PCR after bisulfite treatment of cfDNA isolated in this manner. Hence, electrophoretic separation of cfDNA allows removal of contamination by cellular DNA and reliable analysis of specific DNA methylation patterns for diagnostic applications.

Bisulfite sequencing analysis of the LINE-1 DNA methylation patterns in cellular DNA showed 62% methylated CpG dinucleotides in the younger and 50% methylated CpGs in the older individuals, respectively (Fig. 3A). This result appears relatively consistent with the MS-PCR result (Fig. 1A/B). Of note, the amplified sequences of the older individuals had 16% CpGs with a technically undefined methylation status, more than in the younger cohort with only 13% undefined CpGs (Fig. 3A).

The cfDNA methylation status in young individuals (Fig. 3B) resembled that of cellular DNA. Importantly, the methylation grade of cfDNA in older individuals was distinctly lower, namely 20% vs. 68% (Fig. 3B). In addition, not a single sequence among the cloned LINE-1 amplicons exhibited dense methylation compared to many sequences in the younger cohort (Fig. 3B). A detailed comparison of the altered methylated CpG positions between younger and older persons (Fig. 3C) identified the most differentially methylated positions allowing to optimize primer design in order to detect these differences most efficiently for monitoring of aging. As stated previously, we consider such detailed analyses as a general epigenetic methodological strategy for any genomic region of diagnostic relevance and a prerequisite for the development of efficiently interrogating MS-PCR analyses. Of note, recently it has been demonstrated that individual LINE-1 CpGs exhibit different levels of methylation in different healthy tissues and in specific tumors underlying the importance of this strategy to reveal the exact CpG methylation pattern in each case^38^.

An interesting point is the origin of hypomethylated cfDNA in the peripheral blood of older individuals. There are several possible explanations. For instance, reactive oxygen species (ROS) have been implicated in cancer and ageing and ROS-induced oxidized DNA lesions, such as 8-hydroxy-2′-deoxyguanosine (8-OHdG) in CpG-dinucleotides, have been shown to strongly inhibit methylation of adjacent cytosine residues^39^. Recently, it has been reported that LINE-1 elements become transcriptionally derepressed also during cellular senescence. The proposed mechanism is a deregulation of the repressors RB1, FOXA1 and TREX1 that relieves LINE-1 from epigenetic repression, activate their promoters and compromise LINE-1 cDNA removal, respectively^40^. Thus it may be hypothesized that aged and senescent cells somehow leak DNA into circulation. In addition, current evidence supports the view that apoptosis may be a major source of cfDNA release^26^. Since LINE-1 hypomethylation and consequent reactivation may severely harm the genomic and functional integrity of a cell they could actually contribute to apoptosis or senescence. Exciting recent evidence that cfDNA is predominantly composed of LINE-1 elements^18^ even suggest the explanation that increasing LINE-1 hypomethylation and retrotransposition activity may contribute to apoptosis as well as the release of cfDNA enriched in hypomethylated LINE-1 sequences. If this idea is correct, the increase in hypomethylated LINE-1 DNA in cfDNA may not only represent a suitable biomarker of human aging, but may also reflect an increasing rate of apoptotic events associated with the deterioration of genomic and epigenetic integrity of cells of various tissues, like the immune and hematopoietic systems, the vascular endothelial coating and the liver. Since these changes might partly result from our life-style but are considered to be reversible, one might speculated that this biomarker would in addition allow health monitoring.

One limitation of our methodical approach is that it does not depict which individual LINE-1 elements are subject to hypomethylation in aging. A further question is to which extent the changes in LINE-1 in aging resemble those in cancer. Future research should therefore assess potential relations and differences of the spectra of hypomethylated LINE-1 retrotransposons in aging and cancer.

LINE-1 hypomethylation occurs in a broad variety of different cancers, often at early stages, e.g. in urothelial cancer^15^, but also appears to contribute to cancer progression, especially once the additional cellular defense mechanisms preventing LINE-1 retrotransposition have been overcome. Therefore, we expect that a degree of LINE-1 hypomethylation in cfDNA that is markedly higher than the average value of healthy individuals at a specific age could be indicative of a higher risk of developing or harboring cancer. For assays addressing this issue, it should however also be considered that individual LINE-1 CpGs exhibit different levels of methylation in different healthy tissues and in specific tumors^38^. In summary, thus, LINE-1 hypomethylation alone or in combination with other epigenetic markers could be helpful to identify individuals at risk for cancer. These points need to be specifically addressed by further studies.

Finally, our ELISA data shown in Fig. 4 do not reveal significant differences in LINE-1 protein expression in peripheral blood between younger and older people. This may be due to the insufficient sensitivity of this technique to detect very low concentrations of free ORF-1p in plasma. Like for LINE-1 methylation in cellular and cfDNA, it would be interesting to investigate LINE-1 protein expression in the plasma of advanced age individuals over 70 years with and without cancer. This may furthermore require separating apoptotic cells from leukocytes and erythrocyte progenitors.

## Material and methods

### Blood samples

All methods were carried out in accordance with relevant guidelines and regulations. We confirm that the experimental protocols were approved, informed consent has been obtained from the participants and an appropriate ethics vote was granted by the ethics commission of the medical faculty of the Heinrich-Heine University Düsseldorf, No. 2018–61. This study was carried out with blood samples of 97 healthy donors from a German population, aged between 19 and 73 years, with a mean age of 40 ± 14.63 (SD) years, of which 46 were male and 51 female. The samples were collected and provided by the University Hospital Düsseldorf blood preservation service. 7 ml blood was collected by venous phlebotomy in EDTA tubes and centrifuged for 10 min at 3600 rpm. After centrifugation, buffy coat and plasma were extracted, coded, frozen and stored at -20 °C until DNA extraction.

### Cellular and cfDNA isolation and bisulfite conversion

Cellular DNA isolation was performed using the QiAamp DNA Blood Mini Kit (Qiagen, Hilden, Germany). CfDNA Isolation from blood plasma was carried out by usingQiAamp DNA Blood Mini Kit (Qiagen, Hilden, Germany), PME free-circulating DNA Extraction Kit (Analytik Jena, Jena, Germany), Quick-cfDNA Serum & Plasma Kit (ZymoResearch, Irvine, CA, USA) and QIAamp MinElute ccfDNA Kit (Qiagen, Hilden, Germany) by following the appropriate manuals. Reproducibly, no cellular DNA contamination was detected on conventional ethidium bromide stained agarose gels (Fig. 5) only by using the QIAamp MinElute ccfDNA Kit (lanes 8/9).

**Figure 5:** Cellular and cfDNA isolation using various commercially available kits. Lane 1: genomic DNA by QiAamp DNA Blood Mini Kit (kit **A**). Lane 2/3: cfDNA by QiAamp DNA Blood Mini Kit (kit A). Lane 4/5: cfDNA by PME free-circulating DNA Extraction Kit (kit **B**). Lane 6/7: cfDNA by Quick-cfDNA Serum & Plasma Kit (kit **C**). Lane 8/9: cfDNA by QIAamp MinElute ccfDNA Kit (kit **D**).

In brief, cell lysis for cellular DNA was carried out at 56 °C for 30 min and the QIAGEN mini columns were incubated for 5 min at room temperature after addition of 35 µl elution buffer AE. The average amount of cellular DNA derived from a single blood sample of 200 µl was 50–240 ng and of cfDNA from a single blood plasma sample was 3 ng. For bisulfite conversion 100 ng cellular DNA, 3 ng of cfDNA and combined multiples of 3 ng were used. Bisulfite conversion was carried out with the EpiTectBisulfite Kit (Qiagen, Hilden, Germany).

### Relative quantification of LINE-1 methylation in cellular and cell-free DNA

Bisulfite-treated DNA served as template for amplification of methylated LINE-1 promotor sequences in a normalized real-time MS-PCR for genetically imbalanced DNA specimens as described^15,17,22,44^. Quantification was done using StepOne Plus Real Time PCR System (Applied Biosystems, Foster City, United States of America) with the following primers for sL1met: 5′-GCGCGAGTCGAAGTAGGGC-3′; asL1met:5′-CTCCGACCAAATATAAAATATAATCTCG-3′. Amplification of an adjacent region without CpGs was used to normalize the amount of LINE-1 methylation. The primers used for reference amplification were for sLcontrol: 5′-AGGTTTTATTTTTGGGGGTAGGGTATA-3′; asL1control:5′-CCCCTACTAAAAAATACCTCCCAATTAAAC-3′^15^.

The following annealing temperatures were chosen: L1met: 61 °C; L1control: 58 °C. The amplification conditions were denaturation at 95 °C for 10 min, followed by 40 cycles of 95 °C for 30 s, TM for 40 s, and 72 °C for 15 s. All reactions were run in triplicates on a Step One Plus Real-Time PCR System (Thermo Fisher Scientific, Massachusetts, USA). Relative differences in DNA methylation were calculated by the ΔΔCt-method.

### Bisulfite genomic sequencing and nested MSPCR

For bisulfite sequencing of the LINE-1 promoter region fragment 8 cfDNA samples from individuals aged 21–29 years and 8 cfDNA samples from individuals aged 50–58 years were combined and mixed. Electrophoretic separation was performed on 1.0–1.2% agarose gels to separate cfDNA fragments in the range between few hundred and 10,000 base pairs. It has been reported that a clear discrimination of apoptotic and necrotic plasma DNA is possible by gel electrophoresis where multiples of 180-bp fragments are thought to originate in apoptotic DNA^41^ and only 0.06% to 0.3% of the cfDNA fragments are longer than 1000 bp^42^. These could originate from cells dying via necrosis. The following primers were used: sLINEkonv1Ampl: 5′-GGT TTA TTT TAT TAGGGA GTG TTA G-3′ and asLINEkonv1Ampl: 5′-ACA AAA ACA AAC AAA CCTCC-3′^17^.

The amplification conditions were denaturation at 95̊°C for 13 min, followed by 35 cycles of 95 °C for 50 s, 51 °C for 45 s, and 72 °C for 30 s. We used 2 µl bisulfite-converted DNA, a 200 μM dNTP mix solution (Promega), 10 pm of each primer and 1.5 units of HotStarTaq DNA Polymerase (Qiagen) per reaction. The amplification product was 436 bp in size. The TA Cloning Kit (Invitrogen) was used for cloning of the amplification products according to the manufacturer’s instructions. Sequence evaluation was performed with the BigDye Terminator Cycle Sequencing Kit (Applied Biosystems) on a DNA analyzer 3700 (Applied Biosystems) using the M13-as primer. On average 30 clones were sequenced to obtain the representative methylation profile of one mixed sample^17,21^. All sequences were aligned using CLUSTLW from the Kyoto University Bioinformatics Center onhttp://www.genome.jp/tools/clustalw/ and all methylated CpGs were manually counted for every single CpG position. For nested PCR amplification of *OR53J3* the following primers were used: Forward 1: 5′-GTG TTG GTG GGT ATT AGT ATG TGT-3′, forward 2: 5′-TGG TGG GTA TTA GTA TGT GTA TTG-3′, reverse1 5′-AAA AAA CAC AAATAA CTC CAA CAT-3′. First round conventional MS-PCR amplification was run for 20 cycles. The second round amplification was then run using a 1:20 dilution for additional 30 cycles at 47 °C to obtain a 334 bp amplicon.

### Enzyme-linked immunosorbent assay, ELISA

The detection of ORF-1 protein in young and old probands was done by sandwich ELISA (Enzyme-linked Immunosorbent Assay). Four times each, 3 different blood plasma samples of individuals aged between 19 and 23 years (young) and 3 different blood plasma samples of individuals aged between 58 and 73 years (old) were measured in triplicates and compared. The assay was performed according to the ELISA technical guide by Thermo Fisher Scientific. We used monoclonal mouse-anti-LINE-1-ORF1, 4H1, MABC1152 (Merck Millipore) as a primary antibody. The polyclonal antibody rabbit anti-Human L1RE1MBS9429742 (BIOZOL) was chosen as the secondary antibody. This secondary antibody was linked with HRP enzyme using EZ-Links Plus Activated Peroxidase Kit (Thermo Fischer Scientific). For the ELISA assay we used 12 µg/ml of each antibody for each well. Protein lysates of the cell line HT-1376 (40 µg), originally isolated from a high grade urothelial cancer of a 58 years old female patient^43^ and kindly provided by the DSMZ (Braunschweig, Germany), which is markedly hypomethylated and known to express LINE-1 ORF1p, and primary urothelium (40 µg), kindly provided by Dr. Michèle J. Hoffmann, Düsseldorf, were chosen as positive and negative references, respectively. The volume of each single blood plasma sample was 50 µl in each well. All buffers needed were provided by the Support Pack Plus Kit (Thermo Fisher Scientific). Finally, the absorbance was measured at 450 nm.

## Supplementary information

Supplementary Information 1.
